# Corrosion Resistance of 3D-Printed Titanium Alloy Ti64-ELI Parts for Dental Application

**DOI:** 10.1155/2022/1804417

**Published:** 2022-04-16

**Authors:** L. Lebea, H. M. Ngwangwa, D. A. Desai, F. Nemavhola

**Affiliations:** ^1^Department of Mechanical and Mechatronic Engineering, Tshwane University of Technology, South Africa; ^2^Unisa Biomechanics Research Group, Department of Mechanical Engineering, University of South Africa, South Africa

## Abstract

Corrosion in the human body can cause materials to change structurally and release undesirable products that may bring about complications such as toxicity and inflammation. These may jeopardize the mechanical stability of prostheses. The purpose of this study was to evaluate the effect of solutions (Ringer's and table salt [NaCl]) and immersion periods on 3D-printed titanium alloy Ti64-ELI samples and the changes in mechanical properties before and after corrosion testing. The microstructure of prepared samples was analyzed, and the formation of *α*- and *β*-phases was studied. During testing, the *β*-phases showed up as white, and the *α*-phases presented as dark. In both, corrosion by pitting was observed after corrosion analysis. The results show that, by comparing NaCl and Ringer's, the *E*_corr_ of the solutions increased by 0.8 V and the *I*_corr_ decreased by an order of magnitude. It was observed that the weight loss in the solutions will lead to dental implant instability and will cause failure.

## 1. Introduction

Titanium (Ti) and titanium alloys are broadly used as contender substances for biomedical implants [1]. Despite their satisfying biocompatibility and good corrosion resistance, these materials still corrode after implantation in biological mediums [2]. An acidic environment, masticatory forces, chlorine presence, and fluoride content all play a role in corrosion. Hank's balanced salt solutions, which can be used to simulate the corrosive environments in the bodies of living organisms, are often used to analyze such corrosion behavior [3, 4]. Several studies have been undertaken in this regard [5–7].

These studies have shown that corrosion by pitting on commercially pure titanium resulted from fluoride ion activity [8]. Ringer's solution was used to demonstrate the corrosion behavior of Ti-Al_2_O_3_, and scanning electron microscope (SEM) images of the samples after prolonged immersion revealed both corroded regions and deposition zones on surfaces [9]. However, the corrosion assessment of 3D-printed material in a controlled environment is still lacking. Additive manufacturing is poised to bring about a revolution in the way products are designed and manufactured [10]. It is therefore of paramount importance that the mechanical properties of additively manufactured specimens be evaluated.

The microstructure and hardness of two titanium alloys have been assessed, and micro- and macrohardness data revealed the Ti–6Al–4V alloy to be harder than its commercially pure (grade 2) counterpart [11]. The Vickers hardness method was used to test a titanium alloy Ti-6Al-4V specimen manufactured by selective laser melting [12]. The results showed a maximum hardness value (HV) of 449.60 and a minimum HV of 380.70. The purpose of this study was to evaluate the effect of solutions (Ringer's and table salt [NaCl]) and immersion periods on 3D-printed titanium alloy Ti64-ELI samples and the changes in mechanical properties before and after corrosion testing.

## 2. Materials and Methods

### 2.1. Samples Preparation

The titanium alloy Ti64-ELI (extralow interstitials) samples utilized for this study are measured 10 × 10 × 2 mm in size. The chemical composition of Ti64-ELI powder is given in Table 1. The 3D-printed samples were washed with distilled water. The mass of all specimens was registered and specified accordingly. A 3.65% NaCl solution and a Ringer's solution were prepared to serve as the corrosive mediums. The solutions (100 ml in all each) were prepared for all corrosion and mass-loss measurements. Immersion and polarization tests were carried out at a temperature of 30°C.

### 2.2. Linear Polarization Resistance

Polarization testing was carried out using an autolab potentiostat instrument with Nova 2.1 software. The system involved three electrodes connected to the equipment. The 3D-printed titanium alloy samples served as the working electrodes. The samples were connected to the equipment and set in beakers, each containing 100 ml of the electrolyte solutions. Potentiodynamic polarization versus open-circuit potential (OCP) curves were obtained from the potential of -1.6 V to 1.6 V at a scan rate of 0.005 m/s. The working electrodes were dipped into the electrolyte solutions (3.65% NaCl solution and a Ringer's solution) for 10 minutes to accomplish the steady-state potential, and the outcomes were recorded. The polarization potential (Ecorr) and current density (jcorr) data were estimated from Tafel plots.

### 2.3. Weight Loss Experiment (Immersion Test)

The 3D-printed titanium alloy samples with dimensions of 10 × 10 × 2 mm were prepared, rinsed with distilled water, and allowed to dry. The precleaned and weighed samples were suspended in beakers containing the NaCl and Ringer's test solutions using glass hooks and rods. The beakers were covered with foil to avoid evaporation during the experiment (Figure 1). The tests were conducted in conditions of total immersion in the solutions. Immersion times varied from one to five days (120 hours). The samples were retrieved from the test solutions every 24 hours, appropriately cleaned, dried, and re-weighed. The weight loss was taken to be the difference between the weight of the samples at a given time and their initial weight. The corrosion rate (*R*) values were obtained by applying the following equation:

(1) $$\begin{array}{c} R=\frac{87.6W}{\text{DAT}}, \end{array}$$

where *W* is the weight loss in milligrams, *D* is the density in g/cm^2^, *A* is the area in cm^2^, and *T* is the time of exposure in hours. The solution efficiency percentage was calculated from the following relationship:

(2) $$\begin{array}{c} \eta =\left(\frac{W_{1}-W_{2}}{W_{1}}\right), \end{array}$$

where *W*_1_ and *W*_2_ are the weight loss in the absence and presence of solutions. The efficiency percentage was calculated for both solutions every 24 hours during the experiment.

### 2.4. Hardness Test Experiment

In this study, a LHBRV-187.5D digital Brinell Rockwell & Vickers hardness tester using an indentation load of 150 kg and a dwell time of 10 seconds was used to measure the hardness of the samples. At least three indents were made across the surfaces of each test specimen. Eighteen specimens were tested overall. Six specimens where tested in each solution before corrosion. The average of each group was computed and used to plot the graphs (Figure 2). The Vickers hardness value (HV) is the ratio of applied load to the surface area of the indent [11].

### 2.5. Microstructure Analysis

The microstructural morphologies of the titanium alloy samples before and after the corrosion experiments were determined with a Zeiss Crossbeam 340 SEM and energy dispersive spectroscopy (EDS) material mapping. Before light microscopy observation, Kroll's reagent was prepared with 100 ml distilled water, 23 ml hydrofluoric acid, and 46 ml nitric acid in accordance with Struers Application Notes on the metallographic preparation of titanium. The samples were etched for 10 to 15 seconds, sprinkled with acetone, rinsed with clean tap water, and dried. The microstructures of all recorded samples were observed under an Olympus BX51M light microscope.

## 3. Results and Discussion

### 3.1. Linear Polarization

Table 2 shows the potentiodynamic polarization data of immersion in the NaCl and Ringer's solutions, respectively. The equivalent polarization curve is shown in Figures 3(a) and 3(b). The jcorr was obtained using Tafel extrapolation of the current potential line. The values of the corrosion rate (Cr) and polarization potential (Pr) were also generated from the Tafel curve.

#### 3.1.1. Polarization Data (NaCl and Ringer's Solution)

The corrosion rate is directly related to the density of the corrosion current. Corrosion potential values (*E*_corr_) correspond with corrosion current density, as shown in Table 2. The Ti64-ELI samples recorded significantly lower corrosion rates in the NaCl solution at 1.8938 mm/year, with the rates increasing to 2.8890 mm/year in the Ringer's solution. Conversely, the polarization resistance was at its highest at 1631.1 *Ω* in the NaCl solution and at its lowest at 214.65 *Ω* in the Ringer's solution (see Table 2).

#### 3.1.2. Open-Circuit Potential (OCP) Measurement

OCP is the potential of the working electrode with respect to the reference electrode when the cell has no current or potential. Changes in open-circuit potential lead to polarization. This is due to the current flow through the electrode/electrolyte interface.  Figure 3 shows the open-circuit potential (OCP) vs. time curve of a 3D-printed titanium alloy in NaCl and Ringer's. The analysis of the OCP vs. time curves shows that the samples in both solutions move the steady-state potential toward a more negative path (Figure 3(a)). The OC*P* values for the samples in the Ringer's solution were between -1,62 V and -0.00015 V within the first 7216.87 seconds. This later changed to less negative values between 0.00092 V and 1.38 V. NaCl solution results indicated OCP values of 1.65 V and -0.00076 V within the first 7233.35 seconds, with a recorded maximum of 1.35 V.

The maximum exposure time was 7244.05 seconds in the Ringer's solution and 7246.86 seconds in the NaCl solution (Figure 3(b)). The OCP plots for 3D-printed Ti64 ELI in Ringer's solutions were observed in the positive to negative potential region, whereas that of NaCl solutions were in negative potential region. A more positive corrosion potential is an indication of a more stable oxide film in a particular environment. This indicates that the 3D-printed titanium samples were more resistant to the Ringer's than the NaCl solution that simulates body fluid.

#### 3.1.3. Potentiodynamic Polarization (PDP) Measurement

The PDP test is performed so that the potential of the test sample increases in stages. This causes an oxidation or reduction reaction on the surface of the test material, and as a result, the current is generated. Tafel extrapolation of the current potential line was used to obtain the jcorr. Corrosion current densities and corresponding corrosion potential (*E*_corr_) values are shown in Table 2. The polarization curve was used to determine the corrosion behavior of the NaCl and Ringer's solutions by Tafel slope extrapolation (Figure 4). The results show that, by comparing NaCl and Ringer's, the *E*_corr_ of the solutions increased by 0.8 V, and the *I*_corr_ decreased by an order of magnitude. The polarization resistance of NaCl solutions was eight times as much as that of the Ringer's solutions. The Ringer's solutions were observed to be more towards passive as compared to NaCl solutions which indicate that the sample in Ringer's solutions has a better corrosion resistance.

### 3.2. Weight Loss (Immersion)

The average mass obtained in each condition over time is presented in Table 3. The experimental immersion process continued for five days to obtain a database on corrosion progress. To plot graphical model, corrosion was measured in terms of the percentage of average mass loss of the specimens at 24-hour intervals. The corrosion progress rates and the efficiency of the specimens are calculated using Equations (1) and (2).

Figure 5 compares the corrosion rates over time in Ringer's and NaCl solutions, respectively. It was noted that when the exposure time changed from 24 hours to 120 hours, the samples in the Ringer's solution corroded more than the samples in the NaCl solution. It was furthermore noted that immersion in the Ringer's solution exhibited a higher weight loss (0.040 g) than did immersion in the NaCl solution (0.021 g) and that prolonging the exposure time to 120 hours resulted in increased weight loss in all conditions (Figure 5).

### 3.3. Hardness Test

The results obtained by using the Brinell hardness tester are presented in Figure 2. Six samples were tested, three indents were made across the surface of each specimen, and the machine provided the HVs. The average values were calculated, with results recorded before and after corrosion testing. The graphical representation of hardness testing shows that the mechanical properties of 3D-printed titanium alloy material changed when exposed to the environment in that samples had a higher HV before corrosion than after corrosion. A linear polarization test was carried out using NaCl and Ringer's solutions. Results showed that the Ringer's solution was more corrosive than the NaCl solution, changing the mechanical properties of specimens and reducing their HVs. Furthermore, corrosion over time was determined. Samples were immersed in both solutions for five days. That reflected an aggressive impact of the Ringer's solution on material, resulting in reduced HVs in specimens immersed in the Ringer's solution compared with those immersed in the NaCl solution.

According to another study [11], the maximum HV of a tested titanium sample is 405.94 HV. The deviation in the current study is less than 4.99%, thus reflecting that the values obtained in this study agree strongly with data reported previously. The parts manufactured through the direct metal laser sintering process presented microhardness values of approximately 370 HV (37.7 HRC) due to the presence of *α*'-martensite [13].

### 3.4. Microstructure, SEM and EDS Mapping Analysis

The morphology and thickness of *α* lamellae are important factors, since they influence the mechanical properties of titanium alloys [14]. To understand this morphology, the Ti64-ELI pattern was analyzed by SEM mapping. Figures 6(a)–6(b) present the SEM micrographs of the samples with different titanium content, clearly reflecting the reported lamellar structures.

Figures 6(a)–6(b) reflect the formation of these phases during the current study. The formation of grain boundaries can be seen in Figure 6(a). The formation of Widmanstatten structures, which occur as a result of the cooling rate during solidification, was observed in a previous study [15]. Widmanstatten structures have two phases, namely, an *α*-phase and a *β*-phase. The *β*-phases are reflected as white and the *α*-phases as dark (see Figure 6(b)).

Figures 7(a)–7(d) show the results obtained by way of polarization and immersion tests. The corroded samples were studied under a microscope to determine corrosion by pitting in Ringer's and NaCl solutions, respectively.

The EDS mapping results of the specimens are shown in Figures 8(a) and 8(b). The wt% for the elements obtained from the EDS analysis of the 3D-printed Ti64-ELI specimens were Ti 89.3%, Al 5.6%, and V 5.1% before corrosion and Ti 94.5%, V 4.2%, and Ca 1.3% after corrosion (see Figures 8(a) and 8(b)). The high percentage of Ti indicates that the alloy did not suffer any dissolution. Analysis before and after corrosion testing showed that the atomic percentage of titanium decreased in the NaCl solution but increased after corrosion in the Ringer's solution.

## 4. Conclusion

This study addressed the effect of solutions (Ringer's and NaCl) and immersion periods on 3D-printed Ti64-ELI specimens and the changes in mechanical properties before and after corrosion testing. The outcomes of the study are:

- Immersion testing was performed to calculate the performance efficiency of the solutions, and it was found that the NaCl solution was more efficient than the Ringer's solution
- Polarization testing showed a lower corrosion rate in the NaCl solution at 1.8938 mm/year. The rate increased to 2.8890 mm/year when Ringer's solution was used. Conversely, polarization resistance was at its highest (1631.10 *Ω*) in the NaCl solution and at its lowest (214.65 *Ω*) in the Ringer's solution
- Furthermore, the Ringer's solution was found to be more corrosive than the NaCl solution, and the hardness properties of corroded samples were lower compared with uncorroded samples
- In conclusion, the problem of dental implant corrosion is usually unthinkable until it becomes a personal health problem for most of us; the lost in weight in NaCl and Ringer's solutions could potentially lead to dental implant instability that will eventually cause implant failure

## Figures and Tables

**Figure 1:** Immersion test using NaCl and Ringer's solutions (a) and polarization test (b).

**Figure 2:** Hardness results before and after corrosion testing.

**Figure 3:** Evolution of OCP: (a) potential versus exposure time for NaCl and Ringer's solutions and (b) Current versus exposure time for NaCl and Ringer's solutions.

**Figure 4:** Tafel polarization graphs of 3D-printed samples immersed in NaCl and Ringer's solutions.

**Figure 5:** Weight loss experiment results: corrosion rate versus exposure time and weight loss versus exposure time.

**Figure 6:** Microstructure of 3D-printed dental implant and formation of martensite structure in titanium material. (a) Grain boundaries. (b) Widmanstatten structures with *α*-phase and a *β*-phase.

**Figure 7:** SEM mapping after corrosion: polarization test in NaCl solution (a); polarization test in Ringer's solution (b); immersion test in NaCl solution (c); and immersion test in Ringer's solution (d).

**Figure 8:** EDS mapping elements before corrosion (a) and after corrosion (b).

**Table 1:** Chemical composition of Ti64-LI powder in percentage by weight (wt%).

Al	V	O	N	C	H	Fe	Y	Other elements	Ti
6.50	4.50	0.13	0.05	0.08	0.012	0.25	0.005	0.1	Bal.

**Table 2:** Polarization data for NaCl and Ringer's solutions.

Solutions	*E*_corr_ (*V*)	*I*_corr_ (*A*)	Corrosion rate (mm/year)	Polarization resistance (*Ω*)
NaCl	-0.48588	0.000163	1.8938	1631.10
Ringer's	-1.3226	0.000142	2.889	214.65

**Table 3:** Average mass loss of test specimens over time.

Time	Ringer's	NaCl
	Weight loss	Weight loss
24	0.031	0.011
48	0.034	0.013
72	0.036	0.017
96	0.037	0.020
120	0.040	0.021

## Data Availability

The datasets used and/or analyzed during the study are available from the corresponding author on reasonable request.
